# An Analysis of Antinuclear Thought in William Golding's Literary Works from the Perspective of Ecoenvironmental Psychology: Taking “Lord of the Flies” as an Example

**DOI:** 10.1155/2022/9158030

**Published:** 2022-07-16

**Authors:** Kanshuai Jiang

**Affiliations:** ^1^College of Literature and Journalism, Xiangtan University, Xiangtan 411105, China; ^2^School of Foreign Languages, Hunan University of Humanities, Science and Technology, Loudi 417000, China

## Abstract

In “Lord of the Flies,” William Golding integrates the living conditions of human beings into the relationship of the community of destiny between man and nature and reveals the neglect of ecological morality in the modern Western ethical value system with modernity as the core, showing a postmodern ecological ethics consciousness beyond modernity. The novel embodies the ecological integrity of the nonbinary opposition between man and nature, criticizes anthropocentrism and technological rationality that destroy the ecological integrity, and points out that modern science and technology have led to greater ecological disasters due to the lack of ecological ethics. Ecological morality that respects nature and the harmonious coexistence of man and nature is advocated. The forward-looking ecological ethics consciousness contained in the novel is especially thought-provoking in today's serious ecological problems and lack of ecological ethics. This paper will use ecological psychology as a new interdisciplinary research field to study the relationship between man and nature and open up new horizons and research methods. In this way, we will solve the growing ecological and environmental crisis.

## 1. Introduction

When British writer Golding's famous work “*Lord of the Flies*” came out in 1954, the multifaceted genre of the work was quite uncertain for critics and readers. The novel is written about the encounters of a group of children who escaped into the children's world due to accidental events, which looks very similar to children's literature; because the story takes place on a desert island, it also resembles the desert island adventure novel in the Western literary tradition (the most familiar one). The masterpiece is Defoe's “*Robinson Crusoe*”; the plot is set in the future era of nuclear war, and it is like science fiction. But all of these are nothing more than literary forms that Golding consciously borrowed and adopted for everyone. In this form, writers explore and think about much more serious practical and philosophical issues. People are very prone to emergencies, such as tsunamis, ice and snow disasters, earthquakes, air disasters, terrorist attacks, and other emergencies. At this time, the inner balance will be easily destroyed, psychological disorders will occur, and some negative emotions such as tension, anxiety, fear, depression, and pain will usher in. Psychologists believe that everyone is constantly striving to maintain a state of inner stability in order to bring harmony between themselves and the environment. Therefore how to carry out psychological intervention, psychological adjustment, and psychological counseling, so that these social individuals can get out of the predicament, restore a good ecological subconscious, so as to better adapt to the changes in the external environment, especially how to correctly guide the young generation to treat scientific and technological development rationally, together with adults jointly shouldering due social responsibilities and devoting ourselves to the cause of world peace are topics that we will continue to explore, as shown in Figure 1.

Ecoenvironmental psychology is a new discipline born from the organic integration of ecological psychology and environmental psychology in the context of environmental crisis in the early 21st century. Its source is ecological psychology [1]. Ecopsychology was born in the 1940s. Gestalt psychologist Lewin published “Psychological Ecology” in 1944. The concept of ecology was introduced into psychological research for the first time [2]. Three years later, another psychologist, Wicker, established a field research station for Chinese and Western psychology in a small town in the United States, advocating natural research methods and behavioral background theory, which marked the beginning of the discipline of ecological psychology [3]. The organic integration of this concept with environmental psychology was in the 1980s. In 1987, the American scholar Jacobs put forward a research theory different from traditional psychological experimental methods on the basis of Buck's ecological psychology research, namely, environmental psychology theory, which focuses on human behavior in natural situations [4]. There was a particular emphasis on the detailed and objective psychological description of human natural behavior in the role relationship with the environment. On this basis, the environmental psychologist Bell first put forward the concepts of environmental psychology such as arousal, overload, adaptation level, behavioral restraint, and stress in his book “Environmental Psychology” published in 2001, which created the conditions for the birth of ecoenvironmental psychology [5]. In 2004, the ecological psychologist D.D.N. Winter and others officially clarified the concept of “ecological environmental psychology” in their book “Psychology in Environmental Problems,” which focuses on the study of environmental physical quantities [6]. The relationship between the environment and the psychological quantities of the environment included the relationship between the environment and people's thinking, emotion, will, and personality, as well as the law of the environment's effect on people's psychology and behavior, including the natural environment (such as noise, temperature, wind direction, climate, and air pollution) and social environment (such as personal space, regional ideas, social atmosphere, social culture, and interpersonal relationships) [7]. In addition, the impact of environmental associations on environmental awareness and psychology, as well as the impact of psychological changes in the process of environmental pollution on the way the human body transmits information and behavior, and how people conduct psychological self-regulation under different environmental conditions to adapt and create a kind of the environment conducive to individual development are the main research content of this new discipline [8].

In view of this, it is a beneficial exploration and attempt to introduce this research into the utilization of nuclear technology [9]. Since the discovery of nuclear fission in 1938, the development of nuclear technology has gone through 84 years of development history. The invention of nuclear technology is recognized as one of the greatest technological inventions of the 20th century, because it has greatly changed the course of human history, including the military use of nuclear energy; for example, the US dropped two nuclear weapons on Hiroshima and Nagasaki, Japan, in 1945 [10]. After the atomic bomb, World War II came to an end, and, from the 1960s to the 1990s, the two superpowers, the Soviet Union and the United States, continuously threatened nuclear weapons, which led to a serious threat to world peace and a deepening fear of people [11]. It also includes the civilian development of nuclear energy since the 1950s, which has made an important contribution to effectively alleviating the world energy crisis [12]. However, it should be noted that, due to paralysis, neglect, and natural disasters, nuclear power generation still poses a serious threat to human life and property safety and environmental protection. The nuclear leak from a nuclear power plant shocked the world [13]. Therefore, since the birth of nuclear technology, nuclear technology has been like a sword of Damocles hanging over people's heads from time to time. It requires people to think about its safe use and strengthen prevention. Human psychology and behavior are not only related to sociocultural factors but also related to the natural environment, as well as environmental psychology from the perspective of psychology and behavioral science, to explore the impact of the environment on people's psychology and behavior. Among them, the introduction of ecological and environmental psychology can help people effectively explore the relationship between environmental physical quantities and environmental psychological quantities in the context of the abuse of nuclear technology, so as to better reveal the law of the effect of the damaged environment on human psychology and behavior [14]. In addition, explore what kind of psychological changes environmental changes bring to people and what coping and intervention mechanisms should be adopted to make psychological adjustments so as to better adapt to changes in the external environment [15]. The protection of life and property and the environment has important theoretical guiding significance and great social value [16].

Similarly, some literary works speak about the effect of the environment on people's psychology and the effect on people's behavior; therefore putting ecological environment psychology into literary works for research can not only expand the horizon of literary research but also better explore the depth of the works' thoughts and reflect the educational function of literary works, especially if they are embedded in ecological literary works. This can better reflect the value of this research [17]. Because ecological literature reflects the interaction between man and the natural environment, different interactions between man and nature will have different effects on their respective evolutionary development. Nuclear literature, as shown in Table 1, which belongs to the category of ecological literature, can better reflect this relationship, because the consequences of nuclear science and technology are the greatest and most profound impact on the natural environment in the application of all scientific and technological achievements, especially the abuse of nuclear science and technology with catastrophic consequences [18]. Through these works, they express not only the pain and pity of nuclear victims but also an appeal to human society, calling for peace, calling for humanitarianism, and calling for human reason, which are the common characteristics and cores shown in these works. Therefore, according to the many painful lessons of human history, combined with their own rich imagination and other forms of literary fiction, the works of many writers in the world have revealed this theme.

These works reproduce the huge disasters brought to mankind by various nuclear explosions, nuclear leakage pollution, and the profound thinking they have made. Many writers have even won the Nobel Prize in Literature for this, as shown in Table 2.

These works further highlight the depth of the social reality reflected in ecological literature such as nuclear literature and the urgency of preventing the misuse of nuclear technology. In addition, these works also show the various psychological and behavioral expressions of people after the nuclear war and nuclear leakage accident, as well as the intervention mechanism and psychological adjustment adopted by these social individuals in order to better survive. For the sake of long-term development, Pausewang, a German female writer, from the perspective of ecological subconsciousness, specially explores the various psychological changes that children and adolescents show in the face of nuclear disasters [19], that is to say, in the face of a nuclear disaster, how people should activate their ecological subconscious and awaken the inherent and healthy environmental interaction consciousness within the ecological subconscious and how to search for various psychological therapy aiming to heal the sense of alienation between people, between people and families, and between people and society and cultivate children with a sound scientific and technological ethics and a sense of moral responsibility, so that they will eventually move towards ecological environmental psychological self-maturity, feeling the beautiful life experience of all things in nature and finally combining world peace with personal happiness; this is the original intention of King Bowser. From the perspective of ecological and environmental psychology, taking author William Golding's work “*Lord of the Flies*” as an example, the following will focus on analyzing how the psychology and behavior of adolescents and children are affected after the nuclear disaster and what people do to them. Moderating and intervening mechanisms to understand the writer's intent in writing, the need for warnings about the misuse of nuclear technology, and the need for nuclear safety education, this will play an extremely important role in enlightenment education for the prevention of social risks and the healthy growth of the next generation of human beings.

## 2. The Psychological Impact of the Nuclear Disaster on Social Individuals, Especially Adolescents and Children

Like natural disasters, nuclear disasters also have three characteristics in common: suddenness, unpredictability, and destructiveness [20]. Specifically, when nuclear explosions or nuclear leaks occur, nuclear disasters are often sudden, powerful, and uncontrollable, and they produce huge damage in a very short time and cause chaos and even destruction in the lives of human and other living beings. Unlike natural disasters, nuclear disasters also have their own characteristics, as shown in Figure 2.

Some studies have found that although natural disasters will bring negative effects on people, such as helplessness, pain, sadness, and other emotions, they can also bring many positive effects, such as social and human solidarity, mutual care, and a sense of social belonging. But technological disasters are different. When a nuclear disaster occurs, although society and individuals also show mutual help and care, psychologically and emotionally, they are more manifested as frustration, depression, curse, pain, withdrawal, numbness, anger, despair, and so forth. In addition, in terms of behavior, people often show selfish behaviors such as selfishness, numbness, rejection, and rejection in order to survive, which is very different from the behaviors that people show in natural disasters.

### 2.1. Work Abstract

During a nuclear war in the future years, a group of British children were evacuated to the rear, and the plane was hit by artillery fire over the Pacific Ocean and fell into the sea. The children who survived escaped on a tropical desert island. At first, the blond boy Ralph and the fat boy with glasses nicknamed Piggy established a civilized order. Everyone divided labor and cooperated, lived together according to the rules and regulations, and lit a fire, hoping to be rescued. However, the bad weather, strange and mysterious environment, and terrifying beasts made everyone feel uneasy. According to some clues, they always thought that there were monsters on the island. Gradually, a big boy named Jack started a conflict with Ralph and the others. He advocated wildness, violence, and bloodshed and was unwilling to wait for rescue according to the rules. He succeeded in pulling most people to his side by this means. Simon is the opinionated one among the children, though he was a little absent-minded on the surface. He found out the truth about the legendary monster and *Lord of the Flies* and was about to tell everyone the whole story. The irascible Jack and his gang did not want him to tell anyone about his discovery, so they bludgeoned him to death. Later, Jack's group smashed Piggy to death and set fire to the jungle on the island, launching an island-wide search to hunt down Ralph. Just as Ralph was cornered, a navy ship appeared on the beach. Facing the incarnation of civilization from the adult world, Ralph could not help but burst into tears.

### 2.2. Appreciation of Works

Reading through “*Lord of the Flies*,” it is not difficult to find that although the children are far away on a desert island, they are always shrouded in the huge shadow of the ongoing bloody war in the adult world. They left their parents and relatives and were forced to evacuate their homeland because of the threat of nuclear war; the reason why they set foot on the desert island was the direct result of the ruthless artillery shooting down their landline. Painful experiences and spiritual trauma are deeply embedded in their young minds, which are the psychological reasons why children are restless, nervous, and panicked all day long on the desert island. At the same time, the abnormal and extreme actions of children, such as zealously hunting wild boars in swarms, notwithstanding the curiosity and adventurousness of children, also have the need to satisfy their appetite and seek survival, which is also directly influenced by the behavior of war. Because of this, through bloodthirsty slaughter again and again, hunters have become murderers, companions have become sacrifices, children themselves have become cannibal monsters, Xanadu has become an arena and a morgue, and the world of innocence has become the base of evil. The wreckage of the plane, the corpse of the paratroopers, and the rescued “warship” in the novel remind readers from beginning to end that children on the desert island simply replay the roles that adults have always played in the big world outside. The island is but a microcosm of the real world, and the ominous giant shadow of “*Lord of the Flies*” looms over the entire planet. Thinking of World War II, which just ended, as well as the Korean War and Vietnam War that resurfaced in the 1950s, the meaning of the future world depicted in “*Lord of the Flies*” is quite clear.

Clearly, “*Lord of the Flies*” is essentially a modern fable. Its implication is not only the confrontation between civilization and barbarism in the context of war but also a deep insight into the heart or human nature. People have human nature, human nature has laws, and the essence of the law of human nature is seeking benefits and avoiding harm. It not only ensures the survival and reproduction of human beings but also causes various social chaos. Golding famously argued that the flaws of society should first be attributed to the flaws of human nature, and his most important mission as a writer is to heal “man's astonishing ignorance of his own nature.” Unlike the Chinese who believe that “nature is inherently good,” Golding agrees with most Westerners that human nature is inherently evil. He demanded that his works must be done so that people can face up to “the sad fact of human cruelty and greed.” “*Lord of the Flies*,” like Golding's other works, is also about the “darkness of the human heart.” Golding's view of human nature and his exploration of human nature have profound ideological origins in Western culture. Both Plato and Aristotle expressed the following views in different terms: man is the best among animals, and he may also be the most savage among animals. Golding holds essentially the same view but prefers to reveal the “darkness of the human heart,” pointing to the fragility of civilization. Undoubtedly, this is the result of the repeated impact on the writers' artistic imagination by the constant cruel facts of human social wars in the twentieth century.

The theme of the novel is “the darkness of the heart.” The excerpt of the story is that after Simon found out the truth about *Lord of the Flies* and the monster, he was ready to report to everyone. Jack and his group roasted wild boar on their own site by the coast to eat. Ralph and Piggy came to check what happened, which is shown in Figure 3. It turns into a maddening spree, and Simon is killed as a beast by the deranged children. The theme is divided into two layers the face unfolds, one is the defeat of Ralph and Jack, and the other is the death of Simon.

By this time, Jack had won over most of the children with his fresh, exciting, and lucrative wild boar hunting. Ralph and his faithful companion Piggy are effectively isolated, with boredom and nothing to do to pass the time. When they came to Jack's group, they were devouring roast pork with relish, leaving them both out in the cold. In the face of Jack's public challenge, Ralph reaffirms his position as the leader. But, in the confrontation between the two, most of the children sided with Jack and were no longer willing to obey any rules. Ironically, even Ralph and Piggy themselves could not resist the temptation to eat roast pork. In Jack's provocative “who wants to join my team” over and over again, Ralph was defeated. He wanted to blow the conch shell to hold a meeting, but everyone was reluctant to listen; he proposed to maintain the fire, but no one paid any attention. Pork, which symbolizes sensual needs, finally defeats the conch, which symbolizes the call of the spiritual soul. The question of whether or not to get rescue and escape from the desert island has also become secondary.

Therefore, the novel “*Lord of the Flies*” is actually a record of the destruction of civilization by barbarism, not a paean to civilization over barbarism. The state of innocence, which is not bound by any laws of civilization, is the state of savagery. The only criterion for selecting barbaric state is whether it is beneficial or effective to maintain survival and development, and then continuously, repeatedly, generation after generation, continuously, and effectively maintain the primitive, barbaric, and ignorant state of existence and development. In a state of savagery, what the human heart has is only instinctive desires, and the senses dictate everything. Such a description obviously denies Rousseau's view that “the return of nature will make the noble savages” and also denies the romantic myths that glorify innocence. Although this pessimistic view of “sex is inherently evil” cannot be said to be comprehensive, it has its own profoundness. Although it is possible to view everything in the world, including human beings, optimistically, blind optimists are not necessarily more sober and wiser than serious pessimists. On the contrary, the view of “evil human nature” can remind people to understand themselves more comprehensively, to actively guard against and prevent their own arrogance, and thus be more profound and valuable.

Simon's death has a deeper meaning and is doubly thought-provoking. Before that, Simon had figured out that the legendary *Lord of the Flies* was actually a large group of flies that fell on the pig head that Jack offered to the gods. Ultimately, *Lord of the Flies* was born thanks to people. First, the material conditions that cause this phenomenon are provided by humans. If Jack had not sacrificed such a big pig's head, there would not have been a gathering of flies. Second, after this phenomenon occurs, people do not study the reasons in detail but rather exaggerate it as an evil spirit in imagination or delirium and exaggerate it as the primordial spirit of flies. The latter aspect was also experienced by Simon during the spasms. In the excerpt, we see that Simon further understands what happened to the monster that once shocked everyone—it turned out to be the corpse of a paratrooper bound by a parachute. The corpse and bones of the corpse also had flies gathered, emitting bursts of stench and making irregular movements. All of this confirms what Simon once said: “The real monster is ourselves.” Although this sentence was regarded as a delusional nonsense and was ridiculed by everyone, it was indeed the case.

Simon has reached the realm of truth, that is, can continue to use and utilize the unique superiority of superb consciousness and wisdom, and, under the effective support, guarantee, motivation, and enlightenment of the superiority of consciousness and wisdom, it can continuously maintain the survival and development more. He has discovered that all demons are actually nothing more than man's own demons. But when he overcame his illness, overcame the difficulty of walking, climbed out of the jungle, and was intent on telling everyone the truth he had discovered, tragedy struck: the children, who had fallen into primitive ecstasy by their revelry, saw him as a “monster” and killed him. This dramatic turning point is a metaphor for the deepest darkness in the human heart: people create and release the devil by themselves, but they do not allow others to expose it, and they dare not face the truth.

Therefore, Simon is the only real hero in the novel, who sacrificed his young life to prove the truth. The description of Simon's body flowing into the sea is full of hazy and mysterious poetry. The author deliberately arranged for a strange little silver creature in the ocean to coalesce into a moving light and shadow, surrounding Simon and bordering his body after death with a shining edge. Under the reflection of the starry sky above him, the body itself is also shining silver. Undoubtedly, this is a sacred sea burial for Simon, to prevent his body from falling into the black mouth of *Lord of the Flies*.

## 3. Postdisaster Psychological Intervention and Confidence Recovery Can Help Adolescents and Children Carry Out Psychological Reconstruction

“*Lord of the Flies*” fully shows the characteristics of fables. Behind the blending of realistic scenes and touching brushstrokes, the characters and plots all contain symbolic meanings. For example, Simon can be called a prophet, Ralph represents honesty and integrity, Piggy represents reason, and Jack is the incarnation of the devil; their quarrel and even confrontation symbolize light and darkness, order and chaos, and savagery and civilization struggle. Even the entire world of children on a desert island can be seen as a symbol of humanity in its original state. There, “evil” occupies an absolute dominant position. It gradually diffuses from the depths of the human heart, swallows up the remaining conscience of the human heart with its irresistible power, and finally has the trend of destroying everything, appearing as *Lord of the Flies*. “*Lord of the Flies*” is etymologically traced back to the Hebrew “Baalzebub.” In the “Bible,” “Baal” is the head of all evil and the king of destruction. Therefore, the essence of “evil” in Golding's writings is the instinct of destruction in the impulse of primitive life will. What the novel “*Lord of the Flies*” does is leading us to cast aside the bouquets and veils of romance, to force us to see the bottomless abyss before which we can tremble and mourn, but in the end we must muster up and have the courage to face it and take responsibility.

The novel “*Lord of the Flies*” reflects the epitome of a real small world encountered by adolescents and children in the face of disaster and has commonalities with nuclear strikes. These all reflect various psychological changes in society, environment, and people in the context of nuclear strikes. In particular, looking at these changes from the perspective of the growth of adolescents and children will have an important impact on the formation of their ecological subconscious, their psychological growth, and their behavior.

After a disaster, people suffer from negative emotions such as fear and worry, as well as feelings of helplessness, sadness, and guilt. How to eliminate all kinds of psychological obstacles, restore the inherent and healthy ecological subconsciousness in the heart, and actively and effectively find a cure for the gradual alienation between people, between people and families, and between people and society and finally move towards mental peace, the maturity of the personality and the beautiful life experience can be started from five aspects, as shown in Table 3.

## 4. The Significance of Strengthening Warnings and Safety Education on the Abuse of Nuclear Technology for the Growth of Teenagers and Children

Strengthening warnings and safety education on the abuse of nuclear technology is important for the growth of adolescents and children, as shown in Figure 4.

Although the content of this novel is the depiction of disasters, and the disaster scenes even seem cruel, “cruelty” is not a gimmick that the writer can manage. On the contrary, these “bloody, scorching purple and black” scenes and various psychological activities reflect the writer's well-intentioned warnings, exhortations, and incentives. The purpose of its warning is that the abuse of science and technology that is not constrained by ethics will only bring disaster to mankind and lead mankind to the abyss of eternal redemption; the purpose of its exhortation is more exchanges and cooperation, more love, and more peace in the world. The purpose of motivation is that the next generation should learn from the shortcomings of the previous generation and have good mental thinking; in the course of their growth, children and adolescents are able to carry out a warning effect and take the initiative to undertake the important task of maintaining world peace. Only in this way can human beings develop sustainably, which is the purpose of the writer's creation of this work.

### 4.1. The Relationship between Man and the Environment from the Perspective of Ecological Psychology

From the above novels and the description of the nuclear strike, it can be found that, due to changes in the environment, there are multiple changes in people's psychology, which affect their behavior; therefore, the relationship between human beings and the environment in which they live has always been a debated issue in many disciplines. This question also plagues the field of psychology, with different schools of thought having completely opposing viewpoints. Behaviorism insists on environmental determinism, while psychoanalysis and humanism exaggerate the role of individual internal factors. It is under this background that ecological psychology comes into being. To put it simply, the relationship between people and the environment is a relationship of mutual restraint and interaction. Among them, mutual restraint is reflected in man's dependence on the natural environment. Human beings themselves are the products of the evolution of nature, and the formation and growth of human beings, as well as their various activities, are inseparable from the need for nature and cannot get rid of the constraints of natural laws. It advocates people to establish correct ecological concepts, promotes the harmonious development between man and the environment, and fundamentally solves environmental problems and ecological crises.

In the 1930s, psychologist Lewin proposed a well-known formula for mental behavior: *b* = *f* (p, e), where *b* represents behavior, *f* represents function, *p* represents person, and *e* represents environment. The formula indicates human behavior. It is a function of the interaction between people and their environment; that is, behavior changes with these two factors. The impact of the environment on people is mainly manifested in some aspects shown in Figure 5.

For the psychological value of the ecological environment to people, ecopsychologists believe that, in addition to historical, economic, and aesthetic values, the ecological environment also has psychological values. The psychological value of ecological environment has the value of development, healing, spirituality, and self-satisfaction, among which the psychological value of wilderness is one of the most valuable fields in ecological psychology, by influencing people's psychological nuclear behavior, so as to guide people to make corresponding psychological changes in nuclear actions. Ecopsychology not only believes that nature participates in people's psychological construction and promotes people's “psychological growth” but also reveals that people's psychology and nature have an innate “emotional connection,” that is, “ecological subconsciousness.” With the alienation of man from nature, this subconscious is suppressed, but this “emotion” is a kind of human nature, and man comes from nature; even after man stands up from nature and obtains the certainty of man, man is not beyond nature, and nature is still the foundation of human existence. There is still an instinctive emotional relationship between human beings and nature. As long as a certain situation occurs, it will appear in our hearts.

The influence of ecological environment on human behavior. With the industrialization and modernization of human society, the living environment of human beings, including the physical environment and social environment, has had a huge impact on human psychology and behavior. For example, environmental factors such as noise, crowding, pollution, and abnormal climate have seriously affected people's physical and mental health. Research in environmental psychology has shown that the incidence of major physical and mental diseases in life, such as depression and chronic fatigue syndrome, is positively correlated with the trend of environmental pollution or environmental deterioration.

However, people are not completely at the mercy of the environment, and people's subjective initiative also affects and changes the environment all the time. In the face of nature, human beings regard themselves as the first of all things and strive for the infinite expansion of science and technology and the continuous growth of material production and show the value of their own existence by conquering nature.

## 5. Conclusion

In general, unlike traditional psychology, ecological psychology believes that the relationship between people and the environment is not an antagonistic relationship but a complex unified whole. But ecopsychology sometimes overemphasizes ecocentrism, the identity of man and animal, and ignores the social nature of man and the environment. It fails to recognize that the relationship between man and the environment is mediated by the relationship between human beings.

All in all, ecological psychology is a rapidly developing research field. It acknowledges that human beings are currently facing a serious crisis of the external living environment and at the same time advocates that, due to the long-term separation of human beings from nature, the inner world of human beings is also facing a spiritual crisis. As a new cross-cutting research field, ecological psychology has opened up a new vision and research method for the study of the relationship between man and nature. At present, the social environment is suffering from continuous deterioration, people are actively developing industry and economy at the same time, and the degree of attention to the environment is far from enough; this paper will introduce ecological psychology into social development. With the continuous deepening of its research, it will play an increasingly important role in dealing with the increasingly serious ecological environment crisis effect.

## Figures and Tables

**Figure 1:** Literary form of works.

**Figure 2:** Characteristics of a nuclear disaster.

**Figure 3:** Two levels of thematic expansion.

**Figure 4:** The profound context of the works.

**Figure 5:** The impact of the environment on people.

**Table 1:** “Nuclear” writers and their works.

The originator of nuclear literature, British science fiction writer	Welles	“A Free World” (1914)
Swiss playwright	Dylan Matt	“The Physicist” (1962)
Japanese writer	Ibushi Troji	“Black Rain” (1965)
German writer	Wolf	“Nuclear Accident: A Day in the News” (1988)

**Table 2:** Nobel Prize winners and their “nuclear” works.

Japanese writer	Kenzaburo Oe	“Hiroshima Notes” (1964)
German writer	Glass	“The Mother Mouse” (1986)
Belarusian writer	Alexievich	“Memories of Chernobyl, Oral History of the Nuclear Disaster” (1997)

**Table 3:** Postdisaster psychological intervention and confidence restoration can help adolescents and children in psychological reconstruction.

1	Start with the external environment and find spiritual comfort and spiritual sustenance from the restoration of nature
2	Restoring life order is an important means of treating psychological trauma
3	Reopening schools
4	Unlimited sympathy for crippled children from nuclear strikes
5	Reshape the image of the previous generation, bravely assume social responsibilities,and let the next generation grow up healthily in a peaceful environment

## Data Availability

The labelled dataset used to support the findings of this study is available from the author upon request.
